# MALAT1 promotes gastric adenocarcinoma through the MALAT1/miR-181a-5p/AKT3 axis

This article has been retracted.

**DOI:** 10.1098/rsob.190095

**Published:** 2019-09-04

**Authors:** Zhengmao Lu, Tianhang Luo, Tao Pang, Zongxin Du, Xiaoyi Yin, Hangtian Cui, Guoen Fang, Xuchao Xue

**Affiliations:** 1 Department of General Surgery, Changhai Hospital, the Second Military Medical University, SMMU, No. 168 Changhai Road, Yangpu District, Shanghai 200433, People's Republic of China; 2 The People's Hospital of Gongliu, No. 71 East Ring Road, Gongliu County, Yili 835400, Xingjiang, People's Republic of China

**Keywords:** gastric adenocarcinoma, metastasis-associated lung adenocarcinoma transcript 1 (MALAT1), miR-181a-5p, RAC-γ serine/threonine-specific protein kinase (AKT3) pathway

## Abstract

Gastric adenocarcinoma, which originates from the gastric mucosal epithelium, has the highest incidence among various malignant tumours in China. As a crucial long non-coding RNA, metastasis-associated lung adenocarcinoma transcript 1 (MALAT1) has been suggested to play an important role in many tumours. Here, we aimed to investigate the role and underlying mechanism of MALAT1 in gastric adenocarcinoma. Quantitative reverse transcription polymerase chain reaction was applied to determine the expression levels of MALAT1 in serum and cell lines. A CCK-8 assay and a clonogenic survival assay were used to examine cell proliferation and apoptosis. The protein level of RAC-γ serine/threonine-specific protein kinase (AKT3) was determined by western blot. Our results showed that MALAT1 was highly expressed in the serum of patients with gastric adenocarcinoma and in cell lines. Downregulating MALAT1 inhibited proliferation and promoted apoptosis of MGC-803 cells. In addition, MALAT1 directly targeted and decreased the expression of miR-181a-5p, which in turn upregulated the expression of AKT3. Further, overexpressing miR-181a-5p or directly inhibiting the AKT pathway with the inhibitor ipatasertib exhibited similar effects to MALAT1 knockdown. Our research proposes a novel mechanism where the role of MALAT1 is dependent on the MALAT1/miR-181a-5p/AKT3 axis. MALAT1 competes with AKT3 for miR-181a-5p binding, thereby upregulating the AKT3 protein level and ultimately promoting the growth of gastric adenocarcinoma.

## 1. Introduction

Gastric cancer is a common malignant tumour of the digestive tract, and has a high incidence and mortality in China [1]. Gastric adenocarcinoma is a type of gastric cancer caused by malignant transformation of gastric gland cells [2]. The incidence of gastric adenocarcinoma accounts for 95% of gastric malignancies [3]. Histologically, according to the Lauren classification, gastric adenocarcinoma is generally divided into two types, intestinal and diffuse. Gastric adenocarcinoma tends to invade the stomach wall, penetrate the muscular mucosa and submucosa and then destroy the muscularis propria [4]. However, the aetiology and pathogenesis of gastric adenocarcinoma are still unclear, limiting the efficacy of clinical treatment for patients with gastric adenocarcinoma.

Long non-coding RNA (lncRNA) is a non-coding RNA molecule containing more than 200 nucleotides [5]. Studies have shown that lncRNA is essential in many biological processes including the regulation of the cell cycle and cell differentiation, the dose compensation effect and epigenetic regulation, making it a hot research subject in genetics [6]. In recent years, emerging evidence has shown that lncRNA plays an important role in tumorigenesis and tumour development, including gastric adenocarcinoma [7–10].

Non-coding nuclear-enriched abundant transcript 2 (NEAT2), also called metastasis-associated lung adenocarcinoma transcript 1 (MALAT1), is a crucial lncRNA that functions in many tumour types, including gastric cancer. It has been reported that MALAT1 contributes to non-small cell lung cancer development via modulating the miR-124/STAT3 axis [11]. In addition, MALAT1 induces colon cancer development by regulating the miR-129-5p/HMGB1 axis [12]. Moreover, MALAT1 promotes proliferation and invasion via targeting miR-129-5p in triple-negative breast cancer [13]. Previous studies have demonstrated that MALAT1 could be used as a biomarker for invasion [14] and metastasis [15] of gastric adenocarcinoma. However, the molecular mechanism underlying MALAT1 regulation on gastric adenocarcinoma is not clear enough. Our current work aimed to elucidate a new molecular mechanism for revealing the action of MALAT1 in gastric adenocarcinoma and to provide new targets and ideas for clinical intervention and the treatment of gastric adenocarcinoma.

## 2. Methods

### 2.1. Patients and samples

Serum samples were collected from 70 patients with gastric adenocarcinoma and 70 healthy controls at Changhai Hospital, the Second Military Medical University. Informed consent forms were signed by all participants. This study was approved by Changhai Hospital, the Second Military Medical University.

### 2.2. Cell culture

The gastric adenocarcinoma cell line MGC-803 and immortalized normal gastric epithelial cell line GES-1 were purchased from ATCC. Cells were cultured in Roswell Park Memorial Institute (RPMI) 1640 medium supplemented with 10% fetal bovine serum and 1% P-S solution (Gibco, Grand Island, NY, USA). Cells were maintained at 37°C under 5% CO_2_.

### 2.3. qRT-PCR analysis

Trizol reagent (Invitrogen, Waltham, MA, USA) was applied to extract the total RNA. A reverse transcription kit (Fermentas) was used for cDNA synthesis using approximately 2 µg of RNA as a template. SYBR-Green Master mix (Life Technologies, Pleasanton, CA, USA) was used for quantitative analysis. The following primers were applied: forward primer 5′-GTCAACGGATTTGGTCTGTATT-3′ and reverse primer 5′-AGTCTTCTGGGTGGCAGTGAT-3′ for GAPDH; forward primer 5′-ATGCGAGTTGTTCTCCGTCT-3′ and reverse primer 5′-TATCTGCGGTTTCCTCAAGC-3′ for MALAT1. GAPDH was used as an internal control for mRNA, and U6 snRNA was used as an internal control for lncRNA and micro-RNA (miRNA).

### 2.4. Cell transfection

A Lipofectamine 3000 kit (Invitrogen) was used for all cell transfections according to the manufacturer's instructions. To knock down MALAT1, the two small interfering RNA (siRNA) oligonucleotides targeting MALAT1 and the negative control were purchased from GenePharma (Shanghai, China) and were transfected into MGC-803 cells. The sequences of the targeting MALAT1 were si-RNA1, sense: 5′-CACAGGGAAAGCGAGTGGTTGGTAA-3; antisense: 5′-TTACCAACCACTCGCTTTCCCTGTG-3′; siRNA-2, sense: 5′-GAGGUGUAAAGGGAUUUAUTT-3′; antisense: 5′-AUAAAUCCCUUUACACCUCTT-3′. The working concentration of relative plasmids was 100 nM.

### 2.5. Cell proliferation

The cell proliferation under various conditions was assessed by means of a Cell Counting Kit-8 (CCK-8). A total of 5000 cells per well were planted into a 96-well plate. A microtitre plate reader (Quant BioTek Instruments) was used to measure the optical density at 450 nm.

### 2.6. Clonogenic survival assay

MGC-803 cells with or without siRNA treatment were planted into six-well plates. After 24 h, cells were exposed to radiation at 8 Gy with an average dose rate of 100 cGy min^−1^. Cells were subsequently maintained for two weeks to allow the colonies to grow at 37°C under 5% CO_2_. Colonies containing over 500 cells were selected and counted as clonogenic survivors.

### 2.7. Bioinformatics

The interaction between lncRNA and miRNA was predicted by the online tool http://starbase.sysu.edu.cn/index.php, and the miRNA target prediction was performed by the online tool http://www.targetscan.org/vert_72/.

### 2.8. Dual-luciferase reporter assay

The sequences of miR-181a-5p including the binding sites of MALAT1 and the mutated binding sites were amplified by polymerase chain reaction (PCR) and cloned into a pMIR vector (Promega Corporation, WI, USA) downstream of a *Renilla* luciferase reporter gene to construct a wild-type miR-181a-5p reporter vector (miR-181a-5p-Wt) and a mutant-type miR-181a-5p reporter vector (miR-181a-5p-mut). MGC-803 cells were co-transfected with miR-181a-5p-Wt or miR-181a-5p-mut and MALAT1 or the scramble lncRNA. Twenty-four hours before transfection, cells were incubated in 24-well plates and transfected with the luciferase reporter vectors. The media were replaced 6 h after transfection and cells were lysed 48 h after transfection. A dual-luciferase reporter assay system (Promega, Madison, WI, USA) and Veritas microplate luminometer (Turner Biosystems, Sunnyvale, CA, USA) were used to measure the luciferase activity.

### 2.9. Statistical analyses

Data are presented as the mean ± s.d. SPSS software (v. 16.0) was used for all statistical analyses. One-way analysis of variance (ANOVA) and Student's *t*-tests were applied to evaluate the differences. Spearman's correlation analysis was applied to examine the significance of association between miR-181a-5p and MALAT1. Significant difference was accepted at *p* < 0.05.

## 3. Results

### 3.1. MALAT1 is highly expressed in patients with gastric adenocarcinoma

In order to identify the function of MALAT1 in gastric adenocarcinoma, we first examined the serum levels of MALAT1 in 70 patients with gastric adenocarcinoma and 70 healthy controls by quantitative reverse transcription polymerase chain reaction (qRT-PCR). The clinical parameters between the two groups of samples including age and gender are shown in electronic supplementary material, figure S1. Statistical analysis indicated that the serum levels of MALAT1 were not affected by these parameters (electronic supplementary material, figure S1A–C). Next, our qRT-PCR results showed that MALAT1 was highly expressed in the serum of patients with gastric adenocarcinoma (figure 1*a*). In addition, patients were divided into two groups according to pathological stage. As shown in figure 1*b*, the expression of MALAT1 in the blood samples of patients with higher malignancy (high-grade group) was significantly higher than that in patients with low malignancy (low-grade group). Therefore, we conclude that MALAT1 is highly expressed in patients with gastric adenocarcinoma and correlates with higher malignancy.

**Figure 1.** MALAT1 is upregulated in the serum of patients with gastric adenocarcinoma compared with healthy controls. (*a*) The MALAT1 expression levels in the serum of 70 patients with gastric adenocarcinoma and 70 healthy controls were determined by qRT-PCR. Results are represented as the mean ± s.d. and ***p < 0.001. (*b*) The MALAT1 expression levels in the serum of patients with patients with low-grade (*n* = 37) or high-grade (*n* = 33) gastric adenocarcinoma were determined by qRT-PCR. Results are represented as the mean ± s.d. and ***p < 0.001.

### 3.2. MALAT1 is highly expressed in gastric adenocarcinoma cell lines

We next compared the expression levels of MALAT1 in gastric adenocarcinoma cell line MGC-803 and gastric mucosal epithelial cell line GES-1. The results showed that MALAT1 was highly expressed in MGC-803 (figure 2*a*), which was consistent with the clinical data. Moreover, we also examined the levels of MALAT1 in normal gastric mucosal epithelial cell line RGM-1 and gastric adenocarcinoma cell line NCI-N87. Excessive expression of MALAT1 was observed in MGC-803 and NCI-N87 compared with GES-1 and RGM-1 (electronic supplementary material, figure S2). We then designed the siRNA and identified the efficiency of the siRNA in the MGC-803 cell line. Our data demonstrated that siMALAT1-1 and siMALAT1-2 worked well for subsequent experiments (figure 2*b*).

**Figure 2.** MALAT1 is upregulated in gastric adenocarcinoma cell lines. (*a*) The MALAT1 expression levels in immortalized normal gastric epithelial cell line GES-1 and gastric adenocarcinoma cell line MGC-803 were determined by qRT-PCR. Results are represented as the mean ± s.d. and *n* = 3 independent experiments. ***p < 0.001 compared with the GES-1 cell line. (*b*) The MALAT1 expression levels in MGC-803 cells after knocking down MALAT1 by siRNA were determined by qRT-PCR. Results are represented as the mean ± s.d. and *n* = 3 independent experiments. ^#^*p* > 0.05 and ***p < 0.001 compared with scramble siRNA.

### 3.3. MALAT1 knockdown inhibits cell proliferation and induces apoptosis in MGC-803 cells

To further explore the biological effects of MALAT1 on cell viability, we then examined the proliferation and apoptosis of MGC-803 cells after knocking down MALAT1. The results showed that, after MALAT1 knockdown, the proliferation ability of MGC-803 cells was significantly reduced (figure 3*a*). A clonogenic survival assay was used to assess cell apoptosis in MGC-803 cells exposed to radiation at 8 Gy with an average dose rate of 100 cGy min^−1^. Cells were then cultured to allow colony formation and the number of colonies was counted. The results showed that knockdown of MALAT1 remarkably reduced the colony number compared with the control group (figure 3*b*), indicating that cell apoptosis was increased by MALAT1 depletion.

**Figure 3.** Downregulating MALAT1 in MGC-803 cells reduces cell proliferation and promotes apoptosis. (*a*) Proliferation of MGC-803 cells with or without siRNA treatment for 1, 2, 3, 4 and 5 days was determined by CCK-8 assays. Results are represented as the mean ± s.d. and *n* = 3 independent experiments, ***p < 0.001 compared with the scramble group. (*b*) The survival curve shows the survival rate of MGC-803 cells with or without siRNA treatment for different time as indicated. The survival rate was detected at 0, 2, 4, 6 and 8 days by a clonogenic survival assay. *n* = 3 independent experiments. ***p < 0.001 compared with the scramble group.

### 3.4. miR-181a-5p is a direct target of MALAT1

To further clarify the mechanism of MALAT1, we predicted the possible binding targets of MALAT1 by bioinformatics. Several miRNAs were found, such as miR-6807-3p, miR-217, miR-181a-5p, miR-3690 and miR-942-5p. We examined the expression of the miRNAs above in MGC-803 cells after knocking down MALAT1. Our results revealed that the expression of miR-181a-5p was significantly upregulated in MALAT1 knockdown MGC-803 cells (figure 4*a*), whereas no significant differences were observed in other miRNAs. The predicted binding sequence is shown in figure 4*b*. The sequences of miR-181a-5p including the binding sites of MALAT1 and the mutated binding sites were subsequently subcloned into a pMIR reporter vector to determine if miR-181a-5p was a direct functional target of MALAT1. In MGC-803 cells, the luciferase reporter assay showed a remarkable decrease in luciferase activity when MALAT1 was co-transfected with miR-181a-5p-WT. However, no significant differences were observed when cells were co-transfected with miR-181a-5p-mut and MALAT1 (electronic supplementary material, figure S3A). We next assessed the expression of miR-181a-5p in gastric adenocarcinoma tissues. As shown in figure 4*c*, the levels of miR-181a-5p were remarkably decreased in gastric adenocarcinoma tissues compared with normal tissues. In addition, the expression of miR-181a-5p was negatively correlated with the expression of MALAT1 (figure 4*d*), indicating that MALAT1 is likely to function by directly targeting miR-181a-5p.

**Figure 4.** miR-181a-5p is a direct target of MALAT1 in gastric cancer. (*a*) MGC-803 cells treated with or without siRNA of MALAT1 were lysed and the miRNA levels were determined by qPCR. *n* = 3 independent experiments, data are presented as the mean ± s.d. and ***p < 0.001 compared with the scramble group. (*b*) The schematics show the interaction between hsa-miR-181a-5p and MALAT1. (*c*) The miR-181a-5p expression levels in 70 pairs of gastric adenocarcinoma and corresponding non-tumour normal tissues were determined by qRT-PCR. Results are represented as the mean ± s.d. and ***p < 0.001. (*d*) Spearman's correlation analysis was performed between has-miR-181a-5p and MALAT1 expression levels (*R*^2^ = 0.2083, *p* < 0.001).

### 3.5. MALAT1 upregulates the expression of AKT3 through targeting miR-181a-5p

We further identified that miR-181a-5p and AKT3 could interact in three positions through bioinformatics prediction (figure 5*a*). The sequences of AKT3 including the binding sites of miR-181a-5p and the mutated binding sites were subsequently subcloned into a pMIR reporter vector to determine if AKT3 was a direct functional target of miR-181a-5p. In MGC-803 cells, the luciferase reporter assay showed a remarkable decrease in luciferase activity when miR-181a-5p was co-transfected with AKT3-WT. However, no significant differences were observed when cells were co-transfected with AKT3-mut and miR-181a-5p (electronic supplementary material, figure S3B). Next, we examined the protein levels of AKT3 under various conditions. Our results showed that MGC-803 cells expressed higher levels of AKT3 than GES-1 cells (figure 5*b,c*). In addition, knockdown of MALAT1 by siMALAT1-1 or siMALAT1-2 reduced the expression of AKT3, consistent with the result that overexpression of miR-181a-5p decreased the protein level of AKT3 (figure 5*b,c*). Therefore, our results suggest that MALAT1 upregulates the expression of AKT3 through targeting miR-181a-5p.

**Figure 5.** AKT3 is directly regulated by miR-181a-5p. (*a*) Bioinformatics analysis showed the interaction in three different locations between miR-181a-5p and AKT3. (*b*) The GES-1 and MGC-803 cells were treated as indicated and the protein levels of AKT3 were determined by western blot. *n* = 3 independent experiments and this panel shows one of these repeats. (*c*) Statistics of the relative levels of AKT3 in (*b*). Data are presented as the mean ± s.d. *n* = 3 independent experiments, ***p < 0.001.

### 3.6. The effects of MALAT1 depend on the MALAT1/miR-181a/AKT3 axis

To confirm whether the inhibitory role of MALAT1 relies on the interaction with miR-181a-5p and the AKT3 pathway, we overexpressed miR-181a-5p or directly inhibited the AKT pathway with the inhibitor ipatasertib in MGC-803 cells. Our results showed that both miR-181a-5p and ipatasertib inhibited cell proliferation (figure 6*a*) and increased cell apoptosis (figure 6*b*) in MGC-803 cells, which is consistent with the effects of MALAT1 knockdown. Our data further indicate that MALAT1 competitively binds to miR-181a-5p, making miR-181a-5p unable to bind to AKT3 mRNA, thereby upregulating AKT3 protein levels and ultimately promoting tumour growth.

**Figure 6.** Overexpression of miR-181a-5p or inhibiting the AKT pathway by ipatasertib have the similar effects of knocking down MALAT1 in MGC-803 cells. (*a*) The cell proliferation of MGC-803 cells transfected with miR-181a-5p or treated with ipatasertib (8 nM) for different times as indicated was determined by CCK-8 assays. Results are represented as the mean ± s.d. and *n* = 3 independent experiments, ***p < 0.001 compared with the control group. (*b*) The survival curve of MGC-803 cells transfected with miR-181a-5p or treated with ipatasertib (8 nM) for different times as indicated. The survival rate of the cells was detected at 0, 2, 4, 6 and 8 days by clonogenic survival assay. *n* = 3 independent experiments. **p < 0.01 and ***p < 0.001 compared with the control group.

## 4. Discussion

Gastric cancer is a malignant tumour originating from the gastric mucosa [16]. In China, there are about 680 000 newly diagnosed gastric cancer patients each year, accounting for half of the global cases, and more than 80% of patients with gastric cancer have reached the middle or late stage when they are diagnosed, meaning that the 5-year survival rate falls below 20% [17]. In 2015, for example, about 498 000 Chinese people died of gastric cancer [17]. LncRNA plays a crucial role in many biological processes [18] and is closely related to various diseases including cancer [19]; therefore, it has become a research hotspot in the life sciences field. Emerging evidence has demonstrated that lncRNAs are critical in tumorigenesis, tumour development and metastasis, prognosis and drug resistance of gastric adenocarcinoma [20]. MALAT1 is a widely studied lncRNA which functions in the tumorigenesis and metastasis of gastric adenocarcinoma. Previous studies have proposed that MALAT1 could be used as a novel biomarker for gastric cancer metastasis [15]. Previous studies examining the expression of MALAT1 have focused on cancer tissue samples from patients, and the expression of MALAT1 in serum has never been detected. In the present study, we demonstrate that the expression of MALAT1 was remarkably elevated in the serum of patients with gastric adenocarcinoma. Our data suggest that MALAT1 might be applied as an auxiliary biomarker for early diagnosis of gastric adenocarcinoma.

Recent studies have reported that MALAT1 might act as a promoter for cell proliferation and metastasis of gastric adenocarcinoma cells. A preliminary study examined some potential target proteins of MALAT1, including N-cadherin, CyclinD1 and Bcl-xl, which are required in apoptosis, cell proliferation, movement and invasion [21,22]. Experiments have shown that knockdown of MALAT1 inhibits the expression of Bcl-xl, N-cadherin and CyclinD1 [15]. In our study, we found that knockdown of MALAT1 significantly inhibited cell proliferation and promoted cell apoptosis, which was consistent with the previous results.

It is well known that miR-181a-5p is essential in the development and differentiation of lymphocytes and vascular endothelial cells [23,24]. However, miR-181a-5p is also involved in many cancer types, such as breast cancer [25], hepatocellular carcinoma [26], multiple myeloma [27] and leukaemia [28]. However, contradictory reports on the effects of miR-181a-5p on promoting or inhibiting tumorigenesis in different tumours have not been answered. Previous research has shown that the expression levels of miR-181a-5p are decreased in some cancer types, including leukaemia, oral squamous cell carcinoma and glioma [29–31]. It has been reported that miR-181a-5p suppresses cell proliferation and migration by targeting Prox1 in HGC-27 cells [32]. Thus, miR-181a-5p is generally considered to be a tumour suppressor based on these findings. Consistent with these previous results, we proved that the expression of miR-181a-5p was remarkably increased in MALAT1 knockdown MGC-803 cells. In addition, the expression of miR-181a-5p was significantly decreased in gastric adenocarcinoma tissues compared with normal tissues. Therefore, we further demonstrate that MALAT1 plays its role in gastric adenocarcinoma by targeting tumour suppressor miR-181a-5p.

AKT is a protein involved in the phosphatidylinositol-3 kinase (PI3K) signalling pathway [33]. Previous studies have reported that AKT is overexpressed at the protein or DNA level in breast and gastric cancer [34]. In addition, the overexpression or abnormal activation of AKT could be used as a biomarker for predicting the invasion and metastasis of human gastric adenocarcinoma [35]. Therefore, AKT has been extensively studied as a novel molecular targeted cancer therapeutic agent. Previous studies have proved that the PI3K–AKT–mTOR pathway is excessively activated in various malignancies, leading to abnormal expression of various genes, such as tuberous sclerosis 1 (TSC1), phosphatidylinositol-4,5-bisphosphate 3-kinase catalytic subunit alpha (PIK3CA), human epidermal growth factor receptor 2 (HER2), epidermal growth factor receptor (EGFR), and phosphatase and tensin homologue (PTEN) [36,37]. In gastric cancer, 30–60% of patients exhibit excessive activation of the PI3K–AKT–mTOR signalling pathway, which is derived from the amplifications of AKT, the loss of PTEN, or the mutations and amplifications of PIK3CA [38]. In this paper, we demonstrate that knockdown of MALAT1 or the overexpression of miR-181a-5p both decreased the expression of AKT3. In addition, overexpressing miR-181a-5p or directly inhibiting the AKT pathway with the inhibitor ipatasertib rescued the inhibitory effects of MALAT1 in MGC-803 cells. Our results demonstrate that direct intervention on the miR-181a-5p or AKT pathway exhibited the same effect as intervention of MALAT1, suggesting that intervention at any node on this pathway may be an effective means of intervention in gastric adenocarcinoma.

In conclusion, we propose a novel mechanism that MALAT1 competitively binds to miR-181a-5p, making miR-181a-5p unable to bind to AKT3 mRNA, thereby upregulating AKT3 protein levels and ultimately promoting tumour growth in gastric adenocarcinoma. These findings provide us with new insights and hints for the early diagnosis and intervention of gastric adenocarcinoma.

## Supplementary Material

Supplementary Figures

Reviewer comments

## Data accessibility

This article has no additional data.
